The article "Value of Ultrasonic Image Features in Diagnosis of Perinatal Outcomes of Severe Preeclampsia on account of Deep Learning Algorithm" was retracted in 2023. Reasons: signs of a paper mill; compromised peer review; unreliable results or conclusions.

# Value of Ultrasonic Image Features in Diagnosis of Perinatal Outcomes of Severe Preeclampsia on account of Deep Learning Algorithm

**DOI:** 10.1155/2022/4010339

**Published:** 2022-01-07

**Authors:** Qiang Wang, Dong Liu, Guangheng Liu

**Affiliations:** ^1^Department of Ultrasonography, Yidu Central Hospital of Weifang, Qingzhou, 262500 Shandong, China; ^2^Department of Ultrasonography, Weifang People's Hospital, Weifang, 261041 Shandong, China

## Abstract

This study is aimed at discussing the value of ultrasonic image features in diagnosis of perinatal outcomes of severe preeclampsia on account of deep learning algorithm. 140 pregnant women singleton with severe preeclampsia were selected as the observation group. At the same time, 140 normal singleton pregnant women were selected as the control group. The hemodynamic indexes were detected by color Doppler ultrasound. The CNN algorithm was used to classify ultrasound images of two groups of pregnant women. The differential scanning calorimetry (DSC), mean pixel accuracy (MPA), and mean intersection of union (MIOU) values of CNN algorithm were 0.9410, 0.9228, and 0.8968, respectively. Accuracy, precision, recall, and *F*1-score were 93.44%, 95.13%, 95.09%, and 94.87%, respectively. The differences were statistically significant (*P* < 0.05). Compared with the normal control group, the umbilical artery (UA), uterine artery-systolic/diastolic (UTA-S/D), uterine artery (UTA), and digital video (DV) of pregnant women in the observation group were remarkably increased; the minimum alveolar effective concentration (MCA) of the observation group was obviously lower than the MCA of the control group, and the differences between groups were statistically valid (*P* < 0.05). Logistic regression analysis showed that UA-S/D, UA-resistance index (UA-RI), UTA-S/D, UTA-pulsatility index (UTA-PI), DV-peak velocity index for veins (DV-PVIV), and MCA-S/D were independent risk factors for the outcome of perinatal children with severe preeclampsia. In the perinatal management of severe epilepsy, the combination of the above blood flow indexes to select the appropriate delivery time had positive significance to improve the pregnancy outcome and reduce the perinatal mortality.

## 1. Introduction

Hypertensive disorder of pregnancy (HDP), a pregnancy-specific disease, includes gestational hypertension, pregnancy with chronic hypertension, preeclampsia-eclampsia (PE-E), and chronic hypertension with preeclampsia [1]. Of which, severe preeclampsia is the main cause of fetal preterm birth and neonatal death. At the same time, severe preeclampsia may lead to abruption placentae, dysfunction of all organs, dropsy of serous cavity, cardiovascular, cerebrovascular accidents, and other serious complications [2, 3]. According to gestational age, severe preeclampsia can be divided into the early stage and the late stage clinically. But the gestational age has not yet been determined. For pregnant women with early severe preeclampsia, termination of pregnancy is generally recommended. However, it will increase perinatal unfavorable prognosis and bring about iatrogenic preterm birth and neonatal death [4, 5].

With the continuous improvement of medical treatment, clinically, for pregnant women with early severe preeclampsia, to reduce the incidence of neonates [6], expectant management is used to prolong the gestational age and gain time to promote fetal lung maturation. For pregnant women with late severe preeclampsia, because they are close to their due dates, fetuses are nearing maturity; through standardized treatment, maternal, and newborn babies are less affected by elective termination of pregnancy [7]. The mechanism of severe preeclampsia is still unclear. Currently, there is still no effective intrauterine therapy for treatment. Thus, the recent studies are focused on understanding the growth and development of the fetus in utero, early diagnosis and treatment of intrauterine abnormalities, and effective prediction of perinatal adverse outcomes.

With the continuous development of imaging technology, a noninvasive method, color Doppler ultrasound is widely used in prenatal diagnosis and hemodynamic examination [8]. Color Doppler ultrasound can detect hemodynamic change of maternal umbilical artery (MUA), uterine artery (UA), middle cerebral artery (MCA), and ductus venosus (DV). Pregnant women with early severe preeclampsia usually have spasm of arterioles and vessel walls throughout the body, lumen stenosis, villous retardation, reduced blood flow to the umbilical artery, and increased blood flow resistance. Color Doppler ultrasound can detect that the umbilical artery-systolic/diastolic (UA-S/D) values increased, which affects the normal development of the fetus [9–11]. During clinical diagnosis, the ultrasonic imaging effect is poor because of the inherent patch noise and texture characteristics of ultrasonic instrument. Different medical personnel have strong subjectivity in the diagnosis of fetal ultrasound images; it is also possible to obtain different measurements for the same object. The deep learning algorithm has made remarkable progress in the field of medical image segmentation with the increase of computing power and data volume. Automatic learning of local features and high-level abstract features through multilayer network is superior to traditional manual extraction and prediction [12].

On account of these reasons, in order to achieve accurate prediction of perinatal adverse outcomes of severe preeclampsia epilepsy, ultrasound on account of deep learning algorithm was used to diagnose severe preeclampsia in pregnant women and evaluate its value in perinatal outcomes in this study.

## 2. Materials and Methods

### 2.1. Study Subjects

From January 2019 to January 2021, 140 pregnant women singleton, who were diagnosed severe preeclampsia by hospital, were selected as the observation group. The age ranged from 23 to 37 years old, with an average age of 30.19 ± 4.78 years old, and gestational age ranged from 31 to 41 years old, with an average gestational age of 33.58 ± 3.81 weeks. All pregnant women had regular menstrual cycles, and the last menstrual history was clear. Fetal malformations were excluded and followed up to the end of pregnancy. At the same time, 140 normal single pregnancy pregnant women, who were hospitalized and delivered in the hospital, were selected as the control group. The age ranged from 22 to 38 years old, with an average age of 31.33 ± 3.97 years old, and gestational age ranged from 32 to 41 years old, with an average gestational age of 33.14 ± 4.29 weeks. There were no statistically significant differences in baseline data such as age and gestational age between the two groups, indicating comparability. This study has been approved by the ethics Committee of hospital. All pregnant women and their families were aware of this study and had signed informed consent.

There were four requirements in the inclusion criteria: First, pregnant women met the diagnostic criteria for severe preeclampsia in hypertensive diseases of pregnancy; second, monocyesis; third, complete clinical data of pregnant women; and fourth, pregnant women with no organic cardiovascular diseases, endocrine disorders, and other diseases.

There were three exclusion criteria: first, women carrying multiple pregnancy; second, pregnant women with chronic hypertension, respiratory diseases, urogenital system, and other serious medical and surgical diseases; and third, pregnant women with cognitive dysfunction.

### 2.2. Ultrasonic Examination Methods

Pregnant women took supine position, if necessary, took side position. With detection frequency 3-8 mHz, color Doppler ultrasonic diagnostic instrument was commonly used to observe fetal biparietal diameter, placenta, fetal heart rate, fetal size, amniotic volume, and other fetal intrauterine development once a week. Then, it observed fetal umbilical artery blood flow S/D, pulsatility index (PI), and resistance index (RI). The umbilical artery within 5 cm from the placental attachment was selected as the measurement site, the angle between the sampling line and the umbilical artery was less than 60°, and sampling time did not exceed 1 min. All the above procedures were performed by the same clinician.

### 2.3. Ultrasonic Image Feature Extraction Algorithm Based on CNN Network

The hemodynamic detection on account of color Doppler ultrasound is of great value in predicting perinatal outcome of severe preeclampsia epilepsy. However, low-resolution ultrasound imaging and complex manual interaction lead to low efficiency of clinical examination. On account of convolutional neural networks (CNN), computer-aided pier control system can excavate deeper features of ultrasonic images, reduce the workload of doctors, and improve the efficiency of disease diagnosis.

The CNN network is a deep learning model with multiple hidden layers. It includes an input layer, convolution layer, pooling layer, full connection layer, and output layer. By reducing neuron connection parameters in the network through local perception and weight sharing, the CNN network improves network training speed [13]. A set of original data is input into the convolutional neural network, and the data obtained after the original data is convolved with the convolution kernel is compared with the feature mapping. For a neural network, its calculation equation on the two-dimensional tensor can be expressed as below equation.

(1) $$\begin{array}{c} b\left[\bar{m},\bar{n}\right]=\underset{i}{\sum }\underset{l}{\sum }a\left[\bar{m}+i,\bar{n}+l\right]w\left[i,l\right]. \end{array}$$

In the equation (1), $b\left[\bar{m},\bar{n}\right]$ represented the two-dimensional tensor of the output, $a\left[\bar{m},\bar{n}\right]$ represented the two-dimensional tensor of the input, and *w*[*i*, *l*] represented the weight of the convolution kernel. For a complete CNN, each layer contained several feature images. It was assume that each layer contained $\bar{n}$ convolution kernels, and each convolution kernel was composed of *i* group parameters. Then, the operation of convolution for each layer could be expressed as follows:

(2) $$\begin{array}{c} b_{\bar{n}}^{s}=\overset{A}{\underset{i=1}{\sum }}w_{\bar{n}i}^{s}b_{i}^{s-1}+c_{\bar{n}}^{s}. \end{array}$$

In equation (2), *b*(*s*/*n*) represented the *s*^th^ layer convolution of the *n*^th^ image feature, and *w*(*s*/*ni*) represented the *i*^th^ image *s* − 1 feature of the convolution layer reflected to convolution kernel parameter of the $\bar{n}$ image feature of the *S*^th^ convolution. *b*_*i*_^*s*−1^ represented the *i*^th^ image feature of the *s* − 1 convolution. *c*(*s*/*n*) represented the bias of the $\bar{n}$ feature image of the convolution at the *s* level. Convolution operation was a linear transformation. In order to achieve multilayer nonlinear features, the convolution layer was usually followed by an activation layer, which was used to obtain the nonlinear features of the image through nonlinear mapping of the feature images obtained from the convolution layer. Take the sigmoid function as an example, the following expression is obtained:

(3) $$\begin{array}{c} f\left(a\right)=\frac{1}{e^{-a}+1}. \end{array}$$

The purpose of pooling layer was to use the principle of local correlation of image to conduct subsampling of the feature image after convolution and aggregate statistics of similar features of the feature image to achieve the function of feature secondary extraction to reduce the feature dimension. Pooling operation had invariability to the transformation of feature image, such as expansion, translation, and rotation, while it participates in the design of the network structure to accelerate the operation speed and prevent the 14^th^ overfitting [14].

Average-pooling, maximum-pooling, and brown-pooling are commonly used. Average-pooling is, namely, only averaging the feature points in the neighborhood, and maximum-pooling is used to obtain the maximum of the feature points in the neighborhood. The difference between maximum pooling and average pooling can be observed in Figure 1.

After the original image passes through the convolution layer and pooling layer, the distributed features learned are mapped to the sample marker space through the full connection layer. The full connection layer processes the image information, transforms the two-dimensional feature graph into one-dimensional feature vector, and then carries out the full neural network training after the feature information is summarized. Different from the convolutional layer, the fully connected layer captures the nonlinear relationship between the comprehensive feature information of the convolutional layer and the subsampling layer to learn the feature information, so as to achieve accurate feature classification.

### 2.4. CNN Model Training

CNN could learn a large number of large mapping relations to describe the association between the input and output. In supervised operation, its sample set was composed of vector pairs. However, the CNN network would lose learning ability because all values of the weight matrix are equal [15]. Given a data set with capacity *M*, the overall cost function could be expressed as below equation:

(4) $$\begin{array}{c} J\left(W,x\right)=\left[\frac{1}{m}\overset{m}{\underset{i=1}{\sum }}J\left(W,b;a^{\left(i\right)},b^{\left(i\right)}\right)\right]+\frac{1}{2}\overset{n_{l}}{\underset{l=1}{\sum }}\overset{s_{l}}{\underset{i=1}{\sum }}\overset{s_{l+1}}{\underset{j=1}{\sum }}{\left(w_{ji}^{\left(l\right)}\right)}^{2} \end{array}$$

or

(5) $$\begin{array}{c} J\left(W,y\right)=\left[\frac{1}{m}\overset{m}{\underset{i=1}{\sum }}\left(\frac{1}{2}{\left\|h_{w,b}\left(a^{\left(i\right)}-b^{\left(i\right)}\right)\right\|}^{2}\right)\right]+\frac{1}{2}\overset{n_{l}}{\underset{l=1}{\sum }}\overset{s_{l}}{\underset{i=1}{\sum }}\overset{s_{l+1}}{\underset{j=1}{\sum }}{\left(w_{ji}^{\left(l\right)}\right)}^{2}. \end{array}$$

In equations (4) and (5), *W*, *y* represented the set of weights and biases, respectively, *m* was the sample size, and *a*^(*i*)^, *b*^(*i*)^ represented the input and output of the *i* data. *w*_*ji*_^(*l*)^ was the weight which connected the neuron *i* of *l* − 1 layer and the neuron *l* of *j*, *h*_*w*,y_*a*^(*i*)^ represented the ideal output of the *i* input, *s*_*l*_ represented the number of neurons in the previous layer, *s*_*l*+1_ represented the current number of neurons, and *n*_*l*_ indicated the number of network layers.

In gradient descent, parameters *W*, *y* were updated according to the following equations.

(6) $$\begin{array}{c} w_{ji}^{\left(l\right)}=w_{ji}^{\left(l\right)}-\alpha \frac{\partial J\left(W,y\right)}{\partial w_{ji}^{\left(l\right)}}, \end{array}$$

(7) $$\begin{array}{c} y_{i}^{\left(l\right)}=y_{i}^{\left(l\right)}-\alpha \frac{\partial J\left(W,y\right)}{\partial y_{i}^{\left(l\right)}}. \end{array}$$

In equations (6) and (7), *α* expressed learning rate, partial derivatives by back propagation algorithm. In the calculation of feed-forward conduction, the activation value *L*_2_, *L*_3_, ⋯, *L*_*n*_*l*__ was first obtained according to the forward conduction equation. For each output unit *i* of *n*_*l*_, its residual could be expressed as the following equation:

(8) $$\begin{array}{c} \delta_{i}^{\left(n_{t}\right)}=\frac{\partial }{\partial z_{i}^{\left(n_{t}\right)}}\frac{1}{2}{\left\|b-h_{W,\text{y}}\left(a\right)\right\|}^{2}=-\left(b_{i}-x_{i}^{\left(n_{t}\right)}\right)\cdot f^{\prime }\left(z_{i}^{\left(n_{t}\right)}\right). \end{array}$$

In equation (8), *z*_*i*_^(*n*_*l*_ − 1)^ and *x*_*i*_^(*n*_*l*_)^ indicated parameters set according to the rule. For each layer of *l* = *n*_*l*_ − 1, *n*_*l*_ − 2, *n*_*l*_ − 3, ⋯2, the residual of the *i* node of the *l* layer could be expressed as the following equation:

(9) $$\begin{array}{c} \delta_{i}^{\left(n_{l}\right)}=\frac{\partial }{\partial z_{i}^{\left(n_{l}\right)}}\frac{1}{2}{\left\|y-h_{W,\text{y}}\left(x\right)\right\|}^{2}=-\left(b_{i}-x_{i}^{\left(n_{l}\right)}\right)\cdot f^{\prime }\left(z_{i}^{\left(n_{l}\right)}\right). \end{array}$$

In equation (9), *f*′() was to derivative *f*() with the activation function, *δ*_*i*_^(*n*_*t*_)^ indicated the residual of output unit *i* on the layer *n*_*l*_, and *w*_*ji*_^(*n*_*l*_ − 1)^ indicated the weight of the neurons *i* and *j* which connected the layer *n*_*l*_ − 2 and the layer *n*_*l*_ − 1. Replacing the relation of *n*, *l* in the 9^th^ equation was needed to obtain the following equation:

(10) $$\begin{array}{c} \delta_{i}^{\left(l\right)}=\left(\overset{s_{l}+1}{\underset{j=1}{\sum }}w_{ji}^{\left(l\right)}\delta_{j}^{\left(l+1\right)}\right)f^{\prime }\left(z_{i}^{\left(l\right)}\right). \end{array}$$

Calculating the required partial derivatives was needed by using the following equation:

(11) $$\begin{array}{c} \frac{\partial }{\partial W_{ji}^{\left(l\right)}}J\left(W,y;a,b\right)=x_{j}^{\left(l\right)}\delta_{i}^{\left(l+1\right)}, \end{array}$$

(12) $$\begin{array}{c} \frac{\partial }{\partial y_{i}^{\left(l\right)}}J\left(W,y;a,b\right)=\delta_{i}^{\left(l+1\right)}. \end{array}$$

All of these could be found in Figure 2.

### 2.5. Evaluation Indexes

Using dice similarity coefficient (DSC), average pixel accuracy (MPA), and mean intersection of union (MIOU) could evaluate the region of interest (ROI) difference between clinician manual labeling and algorithmic automatic labeling. Its calculation equation was as follows:

(13) $$\begin{array}{c} \text{DSC}=\frac{2\times \left|S\cap S_{0}\right|}{S_{0}+S}, \end{array}$$

(14) $$\begin{array}{c} \text{MPA}=\left(1-\frac{\left|S_{0}-S\right|}{S_{0}}\right), \end{array}$$

(15) $$\begin{array}{c} \text{MIOU}=\frac{S_{0}\cap S}{S_{0}\cup S}. \end{array}$$

In equations (13), (14), and (15), *S*_0_ represented the ROI manually labeled by the clinician and *S* represented the ROI obtained by automatic segmentation algorithm. Accuracy, precision, recall, and *F*1-score were used to evaluate the classification effect of the algorithm. The calculation equation was as follows:

(16) $$\begin{array}{c} \text{Accuracy}=\frac{\text{TP}+\text{TN}}{\text{TP}+\text{TN}+\text{FN}+\text{FP}}, \end{array}$$

(17) $$\begin{array}{c} \text{Precision}=\frac{\text{TP}}{\text{TP}+\text{FP}}, \end{array}$$

(18) $$\begin{array}{c} \text{Recall}=\frac{\text{TP}}{\text{TP}+\text{FN}}, \end{array}$$

(19) $$\begin{array}{c} F1=2\times \frac{\text{Precision}\times \text{Recall}}{\text{Precision}+\text{Recall}}. \end{array}$$

In equations (16), (17), (18), and (19), true positive (TP) referred to a true positive sample that would predict positive, true negative (TN) represented a negative sample with a negative prediction, true false (FN) represented a positive sample with a negative prediction, and false positive (FP) represented a negative sample with a positive prediction.

### 2.6. Statistical Analysis

SPSS22.0 statistical software was used to process the test data. Mean ± standard deviation of measurement data was indicated by $\bar{x}\pm s$, and count data was indicated by % and examined by *χ*^2^. *P* < 0.05 indicated statistically significant difference.

## 3. Results

### 3.1. Ultrasonic Image Results on account of Deep Learning Algorithm

The key to diagnose perinatal outcome of severe preeclampsia is to recognize the ultrasonic image features. Therefore, accurate and fast extraction of region of interest (ROI) is the key to evaluate the performance of the algorithm. Therefore, the CNN algorithm was used in this study to identify ultrasound images of pregnant women and automatically extract ROI. The network structure of CNN could ensure a certain tolerance when the input data deformation was large. At the same time, we selected representative images and added different types of noise to study the robustness of CNN algorithm against noise. It was found that the CNN algorithm was robust to a certain degree of Gaussian white noise. However, when white Gaussian noise *μ* = 0 and *σ* was too large, ROI extraction might fail, which can be observed in Figure 3.

DSC, MPA, and MIOU were used to objectively evaluate the accuracy of ROI segmentation by different algorithms. Two typical algorithms such as support vector machine (SVM) algorithm and naive Bayes (NB) algorithm were introduced for comparison. The results showed that the DSC, MPA, and MIOU values of CNN were 0.9410, 0.9228, and 0.8968, respectively, which were obviously better than those of SVM and NB, and the differences were statistically significant (*P* < 0.05), which can be observed in Figure 4.

### 3.2. Classification Performance Based on CNN Model

The CNN algorithm was used to classify the ultrasound images of all single pregnancies. The results showed that accuracy (93.44% vs. 88.32% vs. 84.17%), precision (95.13% vs. 90.44% vs. 91.27%), recall (95.09% vs. 88.77% vs. 91.09%) of CNN algorithm, SVM algorithm, NB algorithm, and *F*1-score (94.87% vs. 91.30% vs. 89.61%), and the four indicators of the CNN algorithm were significantly better and the difference was statistically significant (*P* < 0.05), which can be shown in Figure 5.

### 3.3. Relationship between Ultrasonic Blood Flow Parameters and Perinatal Outcome of Severe Preeclampsia

UA-S/D and electronic fetal monitoring (EFM) of pregnant women in the two groups were analyzed. The results showed that 46 pregnant women in the observation group had abnormal UA-S/D and 29 pregnant women had abnormal EFM. There were 12 abnormal UA-S/D and 13 abnormal EFM in the control group. The incidence of abnormal UA-S/D and abnormal EFM in the observation group was higher than that in the control group, and the difference was statistically significant (*P* < 0.05), which can be shown in Figure 6.

Among 140 perinatal children with severe preeclampsia, the gestational age 34 weeks were divided into 48 cases of early severe preeclampsia and 92 cases of late severe preeclampsia. The analysis of perinatal outcomes of two groups showed that the occurrence rate of the small neonatal asphyxia, gestational age, getting into the NICU, and the incidence of intrauterine growth restriction were higher than early perinatal children with severe preeclampsia. The difference was statistically significant (*P* < 0.05), while the incidence of perinatal death was not statistically significant compared to perinatal children with severe preeclampsia (*P* > 0.05). All of these can be observed in Figure 7.

According to the characteristics of ultrasound images of pregnant women, the CNN algorithm was used to divide the blood flow spectrum into two categories: bad outcome and good outcome. The results showed that compared with normal control group, UA-S/D, UA-PI, UA-RI, UTA-S/D, the uterine artery-pulsatility index (UTA-PI), uterine artery-resistance index (UTA-RI), ductus venosus-pulsatility index for veins (DV-PIV), and ductus venosus-peak velocity index for veins (DV-PVIV) in the observation group were significantly increased, and the difference between groups was statistically significant (*P* < 0.05). However, middle cerebral artery-systolic/diastolic (MCA-S/D), middle cerebral artery-pulsatility index (MCA-PI), and middle cerebral artery-resistance index (MCA-RI) in the observation group were significantly lower than those in the control group, with statistical differences between groups (*P* < 0.05). All of these can be observed in Figure 8.

The receiver operating characteristic (ROC) curve of UA-S/D, UA-PI, UA-RI, UA-S/D, UA-PI, UA-RI, DV-PIV, DV-PVIV, MCA-S/D, MCA-PI, and MCA-RI for the diagnosis of severe preeclampsia were drawn, and the area under the curve was calculated. The results showed that UTA-PI has the best diagnostic effect on adverse outcomes of perinatal children with severe preeclampsia, which can be observed in Figure 9.

Taking the outcomes of perinatal children with severe preeclampsia as independent variables and the occurrence of dynamic and venous blood flow parameters as independent variables, logistic regression analysis showed that UA-S/D, UA-RI, UA-S/D, UA-PI, DV-PVIV, and MCA-S/D were independent risk factors for the outcome of perinatal children with severe preeclampsia (Table 1).

## 4. Discussions

Host defence peptide (HDP) can cause hemodynamic changes in pregnant women and is one of the main causes of maternal and infant death. HDP can cause abnormal blood perfusion in important organs, eventually leading to damage or ischemia failure of vital organs such as the heart, brain, kidney, and even involving intrauterine fetuses in severe cases, resulting in perinatal death [10, 16]. Severe preeclampsia is due to insufficient trophoblast infiltration outside the villi of patients, which leads to abnormal development of placental blood vessels in pregnant women and causes placental ischemia and hypoxia. Thus, a large number of vasoactive cytokines enter the blood circulation to induce systemic inflammatory response and result in insufficient blood perfusion in all organs of the body. The placenta, as the most important target organ of severe preeclampsia, has an important influence on the outcomes of perinatal children with severe preeclampsia [17].

Since color Doppler flow in obstetrics was used in obstetric field, the use of color Doppler technology to measure fetal UA, MCA, and other blood flow velocity waveform provided an effective method for monitoring fetal intrauterine safety [18]. Accurate medical image analysis was the key to clinical disease diagnosis. In computer-aided design, traditional machine learning algorithms relied heavily on professional engineering features. Deep learning algorithms represented by CNN have a high application value due to their strong feature learning ability [19]. In this paper, the antinoise performance of the algorithm was proved by artificially adding white Gaussian noise. After adding white Gaussian noise *μ* = 0, *σ* = 0.05, the ROI region extracted had no significant change compared with Figure 3(b), indicating that the CNN algorithm had certain robustness to white Gaussian noise. Using DSC, MPA, and MIOU could objectively and quantitatively evaluate ROI segmentation results. It was found that the segmentation results of the CNN algorithm were closer to those of doctors' manual tracing. However, for some echocardiograms with low SNR, the segmentation results of the CNN algorithm were not accurate enough. Compared with the SVM algorithm and NB algorithm, CNN algorithm had higher accuracy, precision, recall, and *F*1-score, and rarely mi-scores. Its segmentation accuracy could meet clinical requirements.

Studying fetal intrauterine development from the perspective of hemodynamics is an important means of clinical diagnosis of the mother and the fetus. In this study, the blood flow spectrum changes of UA, UTA, DV, and MCA in pregnant women with severe preeclampsia and healthy controls were detected by color Doppler ultrasound, and the diagnostic effect of each hemodynamic parameter on the adverse outcomes of perinatal children with severe preeclampsia was detected by ROC curve. Changes of UA-S/D, UA-PI, and UA-RI could reflect physiological changes of placenta and fetus in pregnant women. UA-S/D, UA-PI, and UA-RI in the adverse outcome group were significantly higher than those in the good outcome group. It was speculated that the reason might be that the vascular lumen stenosis caused by severe preeclampsia led to the decrease of blood flow at the end of UA diastolic stage, and the increase of fetal blood circulation resistance led to the increase of S/D, PI, and RI. UTA is the circulation of blood flow in the uterus and placenta [20]. In this study, it was observed that UTA-S/D, UTA-PI, and UTA-RI were significantly increased in the adverse outcome group. It was speculated that the causes were arterial lumen stenosis leading to increased UTA blood flow resistance in severe preeclampsia, which led to abnormal functions of various body organs in pregnant women, uterine and placental ischemia, hypoxia, fetal respiratory distress, and intrauterine growth restriction.

As a continuation of the main internal carotid artery, MCA played an important role in providing intracranial nutrition to the fetus. During pregnancy, oxygen-rich blood flow in the placenta was transported to the MCA and ultimately supplies brain growth and development [21]. In this study, MCA-S/D, MCA-PI, and MCA-RI in the adverse outcome group were significantly lower than those in the good outcome group. It was speculated that the reason was the decreased placental blood perfusion in severe preeclampsia. In order to ensure the normal fetal blood oxygen supply, the “brain protection effect” reduced cerebrovascular resistance and increased blood flow velocity. DV was a blood vessel from the fetal umbilical portal sinus and inferior vena cava to the right atrium. Abnormal DV could reflect the pressure changes between the fetal UV and right atrium [22]. In this study, it was observed that DV-PIV and DV-PVIV in the adverse outcome group were significantly higher than those in the good outcome group, which was speculated to be caused by the proliferation of smooth muscle cells in the uterine spiral artery of pregnant women in presevere epilepsy, resulting in arterial luminal stenosis, which reduced UTA blood supply, decreased UA blood flow, and increased DV blood flow parameters. Finally, logistic multifactor regression analysis showed that UA-S/D, UA-RI, UA-S/D, UA-PI, DV-PVIV, and MCA-S/D were all independent risk factors for the occurrence of presevere epilepsy. This was similar to the study results of previous studies [23, 24]. These results suggested that ultrasonographic hemodynamic parameters were of great value in predicting the adverse outcomes of perinatal children with severe preeclampsia.

## 5. Conclusions

The accurate and automatic measurement of ultrasonic hemodynamic changes by deep learning technology was of great significance for the auxiliary diagnosis of severe preeclampsia. In this study, the CNN algorithm was used to achieve automatic classification of ultrasound images of severe preeclampsia. Its segmentation accuracy could meet clinical requirements. However, there were still some deficiencies in this study. The CNN algorithm was used to identify target areas, and only supervised training was adopted. Unsupervised training should be tried in the future study in order to ensure the excellent performance of the network.

## Figures and Tables

**Figure 1:** Maximum pooling and average pooling (2 × 2 filters, Stride = 2).

**Figure 2:** CNN network structure.

**Figure 3:** ROI extraction of CNN algorithm.

**Figure 4:** ROI segmentation result evaluation based on different algorithms. Notes: ^∗^comparison with SVM algorithm, *P* < 0.05, and ^#^comparison with NB algorithm, *P* < 0.05.

**Figure 5:** Classification results according to different algorithms. Notes: ^∗^comparison with SVM algorithm, *P* < 0.05, and ^#^comparison with NB algorithm, *P* < 0.05.

**Figure 6:** Comparison of UA-S/D and EFM results between the two groups. Notes: ^∗^ indicated comparison with the control group, *P* < 0.05.

**Figure 7:** Perinatal outcome of severe preeclampsia. Notes: ^∗^comparison with early severe preeclampsia, *P* < 0.05.

**Figure 8:** Comparison of Doppler blood flow indexes between the two groups. Notes: ^∗^comparison with control group, *P* < 0.05.

**Figure 9:** ROC curve analysis results of different hemodynamic parameters.

**Table 1:** Logistic multifactor regression analysis of perinatal children with severe preeclampsia.

Factors	Partial regression coefficient	Wald	*P*	Odds ratio (OR)	95% chemically induced (CI) OR
UA-S/D	0.84	0.091	0.003	1.665	0.915~1.207
UA-RI	0.11	0.317	0.012	1.052	0.733~1.464
UTA-S/D	0.211	0123	0.039	1.023	0.89~1.225
UTA-PI	0.232	0.087	0.000	1.261	0.844~0.927
DV-PVIV	0.415	0.069	0.006	1.514	1.021~1.338
MCA-S/D	0.217	0.074	0.022	1.242	0.989~1.024

## Data Availability

The data used to support the findings of this study are available from the corresponding author upon request.
